# Effect of Anti-Infective Reconstituted Bone Xenograft Combined with External Fixator on Serum CRP and PCT Levels and Prognosis of Patients with Bone Infection after Lower Extremity Long Bone Trauma

**DOI:** 10.1155/2021/5979514

**Published:** 2021-08-30

**Authors:** Fei Wang, Yang Liu, Xiaofeng Qiu, Hao Fei, Wei Liu, Kun Yuan

**Affiliations:** The First People's Hospital of Nantong, The Second Affiliated Hospital of Nantong University, Teaching Hospital Affiliated to Kangda College of Nanjing Medical University, Nantong 226001, Jiangsu, China

## Abstract

Bone infection is one of the common complications of orthopedic surgery. After bone trauma occurs in the human body, the infection of *Staphylococcus aureus* and Gram-negative bacteria into the fracture area can lead to double infection of the soft tissue and bone tissue at the fracture site, leading to a variety of complications, mostly in the lower extremities. Bone infection easily causes bone destruction, bone nonunion, and bone defect, seriously affecting the quality of life of patients. The traditional treatment method of bone infection is to control the infection first and then repair the bone graft, but this method has a long course, poor efficacy, and high disability rate. In this study, anti-infective reconstituted bone xenograft (ARBX) combined with external fixation was used to treat patients with posttraumatic bone infections of the long bones of the lower extremities, to explore its efficacy, and to analyze its effects on serum CRP, PCT levels, and prognosis. Our results showed that ARBX combined with the external fixator had a good effect on the treatment of patients with bone infection after lower extremity long bone trauma, which could effectively enhance the repair and functional recovery of the limb bone, significantly alleviate the infection degree of patients, reduce the inflammatory response of the body, and have a good prognosis.

## 1. Introduction

Posttraumatic bone infection is one of the common serious complications after open fracture or orthopedic surgery open reduction, which is easy to cause bone destruction, bone nonunion, and fracture nonunion [1, 2]. In the acute phase, the intramedullary cavity is the main infection, often accompanied by high fever, chills, and other sepsis symptoms [3, 4]. In the chronic phase, due to necrosis and infection of the skin and muscle around the fracture end, the blood supply is missing, and the fracture end is directly exposed to the air, resulting in drying and necrosis, so that the adjacent granulation tissue cannot be attached [5, 6]. After soft tissue atrophy, the area of osteonecrosis is further expanded, which is easy to cause bone nonunion or bone defect, which seriously affects the quality of life of patients. The traditional treatment method for chronic bone infection in clinical practice is to control the infection and then repair the bone. This method has a long course of treatment, poor efficacy, and high disability rate [7, 8]. Anti-infective reconstituted bone xenograft (ARBX) has a highly effective osteogenic activity, can release antibiotics locally, and also has a strong anti-infection ability [9, 10]. Synchronous bone grafting on the basis of complete removal of infection can effectively treat bone tissue infection. Effective fixation is the basis for enhancing the stability of the broken end after debridement, which is conducive to promoting bone repair. For patients with severe bone infection, there will often be poor soft tissue coverage conditions, and the effect of internal fixation will be affected [11, 12]. Therefore, the external fixator can be used to fix the patient, which is conducive to the treatment of bone infection. The purpose of this study was to explore the efficacy of ARBX combined with external fixators in the treatment of patients with bone infections after trauma to the long bones of the lower extremities and to analyze its effects on the levels of serum C-reactive protein (CRP), procalcitonin (PCT), and prognosis.

## 2. Materials and Methods

### 2.1. Patients

A total of 62 patients with posttraumatic bone infection of the long bones of the lower extremities who were admitted to our hospital from March 2015 to May 2020 were selected as the research objects, including 40 males and 22 females, aged from 26 to 52 years old, with an average age of (40.58 ± 4.62) years old. Inclusion criteria include the following: involve the long bones of the lower extremities and meet the requirements of posttraumatic bone infection; initial onset or nonhealing or recurrence after antibiotic treatment and surgical treatment; and complete clinical data. Exclusion criteria include the following: those with severe organ diseases; those with systemic metabolic diseases; those with long-term infections and skin cancer; those with severe limb nerve damage that require amputation; and those who fell off during the follow-up. All patients were divided into the control group and observation group by the random number table method, with 31 cases in each group. There was no statistically significant difference between the two groups of general information (*p* > 0.05), and they were comparable, as given in Table 1. This study was approved by the ethics committee of our hospital, and the patients and family members gave informed consent and signed an informed consent form.

### 2.2. Treatment Method

Patients in the control group were treated with traditional treatment. For early infected patients, the fracture internal fixation plate did not need to be removed, but the necrotic tissue and new granulation were directly removed, and the unhealthy tissue of the internal fixation plate was treated together. In advanced patients, the fracture is generally healed, and the internal fixation plate is removed to remove the granulation and the necrotic tissue inside and outside the medullary. Autologous bone graft was performed to restore bone continuity after the local infection was effectively controlled. The observation group was treated with ARBX combined with external fixation after the lesion was completely removed. All fixation methods were replaced with external fixation, and different operations and fixation methods were used according to the location and condition: the incision should be made as far as possible to avoid the scar area or from the edge of the flap, reveal the broken ends, remove the fibrous scar tissue and free dead bone at the broken end, open the medullary cavity, and repair the broken end into a plane or trapezoidal shape, which is conducive to the compression of the broken ends. The broken end can be grafted with ARBX alone, autogenous iliac crest graft, or autogenous fibula graft. Depending on the site of infection, osteotomy can be performed in the proximal or distal epiphyseal areas of the femur or tibia. The osteotomy plane is oblique or transverse, and the periosteum is continuous. All femurs were lengthened by stage I bone grafting and external fixator. The osteotomy began to be extended 5–7 days after the osteotomy, 1 mm/d, divided into 4 times, until it reached the predetermined length. Fixation method: cross drill 2 fixed needles (3-4 mm in diameter) into the distal and proximal ends of the femur or tibia and fibula, respectively, connect the half ring, and the needle angle is 20°–40°. Drill another 2 fixation pins near the fracture of the femur or tibia to connect the half ring. After the fixation is completed, confirm again that there is no missing force line. If the foot drop deformity exists at the same time, an external fixator can be used to correct the foot drop, and needles are inserted into the heel bone and the metatarsal to install a half ring. A compression extension device is connected between the half ring and the calf holder, and the postoperative pressure is slowly applied to correct the foot drop.

The fracture sites of both groups were continuously lavage with normal saline after operation, and antibiotics were selected after secretion culture results were obtained. The wound dressing was changed regularly, and needle route nursing was performed. On the 2nd day after operation, the lower limbs started to perform active and passive flexion and extension exercises for each joint. X-ray examinations were performed at 2, 4, 6, 12, 24, and 48 weeks after surgery to observe the soft tissue, nail path, and osteogenesis.

### 2.3. Observation Index

Peripheral blood samples were collected before and 3 months after surgery, respectively, and serum levels of C-reactive protein (CRP) and procalcitonin (PCT) were determined by the enzyme-linked immunosorbent assay. Relevant test kits were purchased from Shanghai Enzyme Link Biotechnology Co., Ltd., and the specific operation methods were strictly in accordance with the instructions. All patients were followed up for 12 months after surgery, and the effects of bone repair and functional recovery in the two groups were evaluated according to the Ilizarov method and Applications Society (ASAMI) classification criteria [13, 14]. Bone repair evaluation includes four items: fracture healing, infection control, force line restoration, and limb length. Evaluation criteria include the following: excellent: fracture healing, no signs of infection after inspection for 3 consecutive months, force line deformity ≤7°, and limb length difference <2.5 cm. Good: the fracture has healed and meets any 2 of the other 3 items. Acceptable: the fracture has healed and meets any of the other 3 items. Poor: nonunion or recurrence of fractures or fracture healing, but the line of force deformity >7°, and the limb length difference >2.5 cm. The evaluation criteria for functional recovery include exercise, claudication, stiffness, reflex sympathetic dystrophy (RSD), and pain. Evaluation criteria include the following: excellent: good activity, no claudication, knee/ankle back extension loss ≤15°, no RSD, and no pain. Good: can be active and meet any 3 of the other 4 items. Acceptable: can be active and meet any 1-2 of the other 4 items. Poor: inability to complete daily activities.

### 2.4. The Definition of Prognostic Adverse Events and Survival Time

The complications and recurrence of the two groups during the follow-up period were recorded. Patients with nonunion, nail tract infection, and other complications were defined as having adverse prognostic events. Survival time was defined as the time from surgery to complications.

### 2.5. Statistical Method

The results of this experiment were statistically analyzed by SPSS 20.0 (SPSS Co., Ltd., Chicago, USA). Count data were expressed by rate, and the chi-square test was used for their comparison between groups. Measurement data were expressed by mean ± standard deviation, and the *t*-test was used for their comparison between groups. The Kaplan–Meier survival curve was used to analyze the difference of postoperative survival between two different treatment methods, and the log-rank test was used for comparison. *P* < 0.05 indicates that the difference is statistically significant.

## 3. Results

### 3.1. Comparison of Serum CRP and PCT Levels before and after Operation between the Two Groups

At 3 months after operation, the serum CRP and PCT levels of the two groups were lower than those before the operation, and the observation group was lower than the control group, and the differences were statistically significant (*p* < 0.05), as shown in Figure 1.

### 3.2. Comparison of Bone Repair between the Two Groups

After 12 months of follow-up, in the control group, 10 cases of bone repair were excellent, 12 cases were good, 6 cases were acceptable, and 3 cases were poor; the excellent and good rate was 70.97%. In the observation group, 18 cases of bone repair were excellent, 10 cases were good, 3 cases were acceptable, and 0 cases were poor; the excellent and good rate was 90.32%. The excellent and good rate of bone repair in the observation group was higher than that in the control group, and the difference was statistically significant (*p* < 0.05), as shown in Figure 2.

### 3.3. Comparison of the Functional Recovery of the Affected Limbs between the Two Groups

After 12 months of follow-up, in the control group, 8 cases of limb function recovery were excellent, 11 cases were good, 8 cases were acceptable, and 4 cases were poor; the excellent and good rate was 61.29%. In the observation group, 14 cases of limb function recovery were excellent, 12 cases were good, 4 cases were acceptable, and 1 case was poor, the excellent and good rate was 83.87%. The excellent and good rate of functional recovery of affected limbs in the observation group was higher than that in the control group, and the difference was statistically significant (*p* < 0.05), as shown in Figure 3.

### 3.4. Comparison of Complications between the Two Groups

During the 12-month follow-up, 4 cases of nonunion occurred in the control group, 5 cases of nail tract infection, the total incidence of complications was 29.03%, and 2 cases of infection recurrence. In the observation group, there was 1 case of nonunion, 2 cases of nail tract infection, the total incidence of complications was 9.68%, and 1 case of infection recurrence. The total incidence of complications in the observation group was lower than that in the control group, and the difference was statistically significant (*p* < 0.05), as shown in Figure 4.

### 3.5. Comparison of Survival Differences between the Two Groups

The median time to complications in the control group was 9.28 months, and the median time to complications in the observation group was 11.05 months. The median time to complications in the observation group was higher than that in the control group, and the difference was statistically significant (*p* < 0.05), as shown in Figure 5.

## 4. Discussion

Bone infection is one of the common complications of orthopedic surgery. After bone trauma occurs in the human body, the infection of *Staphylococcus aureus* and Gram-negative bacteria into the fracture area can lead to double infection of the soft tissue and bone tissue at the fracture site, leading to a variety of complications, mostly in the lower extremities [15, 16]. Bone infection is associated with both orthopedic internal fixation surgery and trauma, and the incidence of posttraumatic bone infection is about 10%, which can seriously affect the life and health of patients, and it is difficult to treat [17]. Traditional treatment typically involves a phased approach, with the infected tissue removed, followed by a second course of bone grafting or internal fixation three to six months after the wound has healed, followed by antibiotic treatment. However, the use cycle of this method is long, which is prone to adverse reactions, and it is difficult to ensure that the concentration of antibiotics meets the antimicrobial standard, leading to the failure of anti-infection [18]. The newly emerging membrane induction technology requires a second surgical treatment, which greatly increases the patient's pain and medical expenses [19]. The microsurgery technique will increase the damage to the donor site, making it unacceptable for some patients [20]. Once improperly handled, the infection recurs, which will lead to failure of implant fixation or bone grafting. Therefore, it is particularly important to further seek more effective treatment methods.

CRP is a protein that rises sharply in the plasma when the body is infected or tissue damaged, and it can clearly reflect the body's inflammatory response state [21–23]. PCT reflects the active degree of systemic inflammatory response, which is usually stable. Relevant studies have shown that the level of PCT in patients with the presence of infection will increase significantly, and it will decrease significantly with the control of the disease, and there is a positive correlation between the level of PCT and the degree of infection [24–26]. The results of this study showed that 3 months after operation, the levels of serum CRP and PCT in both groups were lower than before operation, and the observation group was lower than the control group. It shows that the use of ARBX combined with the external fixator to treat patients with bone infection after long bone trauma of lower extremities can significantly alleviate the patient's infection degree and reduce the body's inflammatory response. Analysis is for the reasons, ARBX could efficiently induce distribution of active at the same time, also can effectively slow release of antibiotics, can make the antibiotics in the local area to maintain 30 d and slow release medium use convenience, can act according to the preoperative patients with bacterial culture and drug susceptibility test results, and the use of effective antibiotics, to avoid the occurrence of the bacterial drug resistance [27, 28].

The results of this study showed that after surgery, the excellent rate of bone repair and functional recovery of affected limbs in the observation group was higher than that in the control group. It shows that the use of ARBX combined with the external fixator to treat patients with bone infection after long bone trauma of lower limbs has a good effect and can effectively enhance the bone repair and function recovery of the affected limb. The reason is that effective bone grafting at broken ends is the key to the treatment of bone nonunion and bone defect. ARBX contains bone morphogenetic protein with highly effective osteogenic activity obtained from bovine cortical bone, supplemented by bovine cancellous bone as the carrier. Bovine cancellous bone has good bone conduction and bone guidance. After deantigen treatment such as degreasing and deproteinization, it is compounded with bone morphogenetic protein. The bone morphogenetic protein can fully release the bone morphogenetic protein and exert the local bone-inducing effect of the bone morphogenetic protein, which is beneficial to the patient's bone repair and the function recovery of the affected limb. Effective fixation is also the key to promote bone repair. The external fixator used in this study was fixed with fine Kirschner wire and needle, which had little impact on the trauma and blood supply of the patients. Moreover, multiplane fixation could be performed according to the condition of the affected limb, which was conducive to the reconstruction of blood circulation between broken ends and the promotion of bone repair. Moreover, the support strength of external fixation frame is large, so patients can carry out functional exercise early, which is conducive to promoting local blood circulation and promoting the functional recovery of the affected limb.

The results of this study showed that the total incidence of complications in the observation group (9.68%) was lower than that in the control group (29.03%), and the median time to complications in the observation group was higher than that in the control group. It shows that the prognosis of patients with bone infection after long bone trauma with ARBX combined with the external fixator is better. The author believes that in the treatment of posttraumatic bone infections of the lower limbs, we can give full play to the advantages of the external fixator. Half needle or fine Kirschner wire can be used for fixation to reduce the impact on local blood supply. At the same time, the skin graft area should be avoided as much as possible. It can make full use of the elastic fixation of the external fixator, and early training of the knee and ankle joints is conducive to the recovery of the function of the affected limb. Effective control of infection is the key to successful surgery. Therefore, it is extremely important to completely remove the infection. The old scar granulation tissue should be removed completely during the operation to avoid increasing the risk of infection.

## 5. Conclusion

ARBX combined with the external fixator has a good efficacy in the treatment of patients with bone infection after lower extremity long bone trauma, which can effectively enhance the bone repair and functional recovery of the affected limb, significantly alleviate the infection degree of patients, reduce the inflammatory response of the body, and have a better prognosis.

## Figures and Tables

**Figure 1:** Comparison of serum CRP and PCT levels before and after operation between the two groups. (a) Comparison of CRP levels between the two groups. (b) Comparison of PCT levels between the two groups. *Note*. Compared with before operation, ^*∗*^*p* < 0.05. Compared with the control group 3 months after surgery, ^#^*p* < 0.05.

**Figure 2:** Comparison of bone repair between the two groups. *Note*. Compared with the control group, ^*∗*^*p* < 0.05.

**Figure 3:** Comparison of the functional recovery of the affected limbs between the two groups. *Note*. Compared with the control group, ^*∗*^*p* < 0.05.

**Figure 4:** Comparison of complications between the two groups. *Note*. Compared with the control group, ^*∗*^*p* < 0.05.

**Figure 5:** Comparison of survival differences between the two groups.

**Table 1:** Comparison of two groups of general information (*n*, mean ± SD).

Clinical information	*n*	Control group	Observation group	*χ*^2^/*t*	*P*
Gender				2.536	0.111
Male	40	23	17		
Female	22	8	14		
Age (year)	62	40.43 ± 4.71	40.73 ± 4.59	0.254	0.8
Cause of injury				1.833	0.399
Traffic injury	32	18	14		
Fall	18	9	9		
Fall from height	12	4	8		
Type of fracture				1.476	0.224
Open fracture	48	26	22		
Closed fracture	14	5	9		
Site of bone infection				0.847	0.655
Femoral shaft	17	10	7		
Tibia shaft	31	15	16		
Bilateral tibial shaft	14	6	8		

## Data Availability

The data used to support the findings of this study are available from the corresponding author upon request.
